The article "Modulation of GABAergic Synaptic Transmission by NMDA Receptors in the Dorsal Horn of the Spinal Cord" was published in 2022. Journal: Front Mol Neurosci.

# Modulation of GABAergic Synaptic Transmission by NMDA Receptors in the Dorsal Horn of the Spinal Cord

**DOI:** 10.3389/fnmol.2022.903087

**Published:** 2022-07-04

**Authors:** Benjamin Leonardon, Lou Cathenaut, Louise Vial-Markiewicz, Sylvain Hugel, Rémy Schlichter, Perrine Inquimbert

**Affiliations:** ^1^Centre National de la Recherche Scientifique, UPR 3212 Institute of Cellular and Integrative Neurosciences, Strasbourg, France; ^2^Université de Strasbourg, Strasbourg, France

**Keywords:** dorsal horn, synaptic inhibition, NMDA receptors, nociception, pain

## Abstract

The dorsal horn (DH) of the spinal cord is an important structure involved in the integration of nociceptive messages. Plastic changes in the properties of neuronal networks in the DH underlie the development of analgesia as well as of hyperalgesia and allodynia in acute and chronic pain states. Two key mechanisms are involved in these chronic pain states: increased electrical activities and glutamate release leading to the recruitment of NMDAr and plastic changes in the synaptic inhibition. Although: (1) the balance between excitation and inhibition is known to play a critical role in the spinal network; and (2) plastic changes in spinal excitation and inhibition have been studied separately, the relationship between these two mechanisms has not been investigated in detail. In the present work, we addressed the role of NMDA receptors in the modulation of GABAergic synaptic transmission in the DH network. Using tight-seal whole-cell recordings on adult mice DH neurons, we characterized the effect of NMDAr activation on inhibitory synaptic transmission and more especially on the GABAergic one. Our results show that, in a subset of neurons recorded in lamina II, NMDAr activation facilitates spontaneous and miniature GABAergic synaptic transmission with a target specificity on GABAergic interneurons. In contrast, NMDA reduced the mean amplitude of evoked GABAergic IPSCs. These results show that NMDAr modulate GABAergic transmission by a presynaptic mechanism of action. Using a pharmacological approach, we investigated the composition of NMDAr involved in this modulation of GABAergic synaptic transmission. We found that the NMDA-induced facilitation was mediated by the activation of NMDAr containing GluN2C/D subunits. Altogether, our results bring new insights on nociceptive information processing in the spinal cord network and plastic changes in synaptic inhibition that could underlie the development and maintenance of chronic pain.

## Introduction

The dorsal horn (DH) of the spinal cord is an important structure involved in the integration and transmission of nociceptive messages from the inner and outer environment. Spinal integration of this information relies on the interplay between different DH neurons forming a complex and functionally plastic neuronal network (Cordero-Erausquin et al., 2016).

The article "Modulation of GABAergic Synaptic Transmission by NMDA Receptors in the Dorsal Horn of the Spinal Cord" was published in 2022. Journal: Front Mol Neurosci.

The DH neuronal network is composed of inhibitory and excitatory interneurons. A fine-tuning of the excitatory/inhibitory balance is crucial in the control of the transmission of nociceptive messages from the DH to the supraspinal structures where it may lead to pain perception. Imbalance between excitation and inhibition in DH networks is known to be one of the mechanisms leading to enhanced pain sensation and underlying the development and maintenance of pathological pain, such as neuropathic pain. Impairment of DH inhibitory synaptic transmission plays a pivotal role in this disruption of the excitation/inhibition balance (Sivilotti and Woolf, 1994; Coull et al., 2003; Harvey et al., 2004; Torsney and MacDermott, 2006). Indeed, pharmacological blockade of ionotropic GABA_A_ and glycine receptors induces thermal hyperalgesia and mechanical allodynia (Beyer et al., 1985; Roberts et al., 1986).

The major excitatory transmitter released by primary afferent fibers is glutamate. Under physiological conditions, fast glutamatergic transmission in the DH is mediated by postsynaptic AMPA receptors (AMPAr). Sustained or repeated afferent fiber stimulation leads to an increased release of glutamate in the DH and consequently to the recruitment of NMDA receptors (NMDAr; Woolf and Thompson, 1991). In the DH, NMDAr activation is critically involved in long-term potentiation of excitatory synapses (Woolf and Salter, 2000; Sandkuhler, 2007; Latremoliere and Woolf, 2009). Moreover activation of presynaptic NMDAr expressed on afferent fiber terminals facilitates glutamate release in the DH (Liu et al., 1994, 1997; Bardoni, 2013) and modulates transmission of nociceptive messages in the spinal cord (Bardoni, 2013; Deng et al., 2019). Interestingly, one study demonstrated that 37% of GABAergic synaptic terminals in the DH of the rat spinal cord expressed NMDAr (Lu et al., 2005), but the subunit composition as well as the role of these presynaptic receptors has not been investigated so far.

Plastic changes in the strength of inhibitory synaptic transmissions play a crucial role in information processing and tuning of neural activity. In several regions of the CNS, activity-dependent long-term plasticities (LTP and LTD) of inhibitory synapses have been described (Kullmann et al., 2012). In the DH, one study has described a heterosynaptic plasticity at GABAergic synapses in lamina I neurons, after activation of metabotropic glutamate receptors (Fenselau et al., 2011) and one recent study described an NMDAr-dependent potentiation of glycinergic synapses (Kloc et al., 2019). In other structures, postsynaptic and presynaptic NMDAr have been shown to be key players in the modulation of GABA release (Glitsch and Marty, 1999; Duguid and Smart, 2004; Crabtree et al., 2013) and in the functional plasticity of inhibitory synapses (Nugent et al., 2007; Mapelli et al., 2016). It is known that changes in spinal inhibition are crucial in the processing of nociceptive information and that NMDAr are activated by an increased activity in the DH network. However, nothing is known about the possibility that activity-dependent modulation at inhibitory synapses engaging NMDAr could take place in the DH.

The article "Modulation of GABAergic Synaptic Transmission by NMDA Receptors in the Dorsal Horn of the Spinal Cord" was published in 2022. Journal: Front Mol Neurosci.

In the present work, we addressed the role of NMDAr in the modulation of GABAergic synaptic transmission in the DH network. Using patch-clamp recordings on adult mice DH neurons, we characterized the effect of NMDAr activation on inhibitory synaptic transmission and more especially on the GABAergic one. Our results indicate that NMDAr activation differentially modulates spontaneous and electrically-evoked GABA release and that this effect targets preferentially GABAergic synapses established with GABAergic interneurons.

## Materials and Methods

### Animals

All procedures were performed in accordance with European directives and were approved by the regional ethics committee and the French Ministry of Agriculture (license No. 2015030911301894). We used C57BL/6j (*n* = 118) and GAD65-eGFP mice (*n* = 28). GAD65-eGFP were obtained from Ferenc Erdelyi and Gabor Szabo (Institute of Experimental Medicine, Budapest) and have been described previously (Cui et al., 2011). The mice were interbred, born and housed in the animal house of the laboratory (Chronobiotron, agreement No. A67-2018-38) at room temperature with a 12 h light/dark cycle and with free access to food and water. Experiments were performed with male adult mice (5–10 weeks old).

### Slice Preparation

Mice were anesthetized by intraperitoneal injection of urethane (1.9 g/kg body weight) prior to realizing a laminectomy. The lumbar spinal cord was removed and immediately immersed in ice-cold sucrose-based artificial cerebrospinal fluid (sACSF) containing in mM: sucrose (252), KCl (2.5), NaCl_2_ (2), MgCl_2_ (2), glucose (10), NaHCO_3_ (26), and NaH_2_PO_4_ (1.25) continuously gassed with carbogen (5% CO_2_ and 95% O_2_). The spinal cord was embedded in agarose (5%) and 300 μm-thick transverse slices were cut through lumbar 3–5 segments using a Leica VT1200S vibratome (Leica Microsystems Inc.). Slices were stored at room temperature (22°C–24°C) in a chamber filled with ACSF containing (in mM): NaCl (126), NaHCO_3_ (26), NaCl_2_ (2), KCl (2.5), NaH_2_PO_4_ (1.25), MgCl_2_ (2), glucose (10), and continuously gassed with carbogen.

The article "Modulation of GABAergic Synaptic Transmission by NMDA Receptors in the Dorsal Horn of the Spinal Cord" was published in 2022. Journal: Front Mol Neurosci.

### Electrophysiology

Slices were transferred to the recording chamber and continuously perfused with oxygenated ACSF. Recordings were performed from lamina II neurons.

Patch pipettes were pulled from borosilicate glass capillaries (1.2 mm o.d. 0.69 mm i.d.; Harvard Apparatus) using a P-1000 puller (Sutter Instruments, Novato, CA, USA) and had final tip resistances between 3 and 6 MΩ. Pipettes were filled with an intracellular solution containing (in mM): CsCl (130), HEPES (10), and MgCl_2_ (2). The intracellular solution had a pH of 7.3 adjusted with CsOH and an osmolarity of 300 mOsm adjusted with sucrose. In these conditions, the theoretical equilibrium potential for Cl^−^ anions was 0 mV.

Whole-cell patch-clamp recordings were performed from neurons identified under visual control using an infrared differential interface contrast optics. Gad65-eGFP neurons were identified using epifluorescent illumination.

Voltage-clamp recordings were performed with an Axopatch 200 B amplifier (Molecular Devices, San Jose, CA) at a holding potential fixed at −60 mV allowing visualization of excitatory postsynaptic currents and inhibitory postsynaptic currents (EPSCs; IPSCs) as inward currents. Recordings were low-pass filtered (5 kHz) and acquired with Clampex software (Molecular Devices, San Jose, USA). Current traces were digitized (10 kHz) and stored on the hard drive of a personal computer. All experiments were performed at room temperature (22°C–24°C).

Paired-pulse ratio experiments were performed by stimulation of a presynaptic neuron with a 0.25 mA current injection with an extracellular electrode filled with ACSF.

The stimulation was performed as described in Cathenaut et al by applying current steps (0.25 ms; 0.10–0.40 mA) through a patch pipette filled with ACSF (Cathenaut et al., 2022). This stimulation electrode was placed at 20–150 μm from the cell body of the recorded neuron. For each recorded neuron, the lowest amplitude of stimulation evoking IPSCs was determined and was increased by 0.05 mA to evoke IPSCs for each stimulation applied. Synaptic contacts were identified as monosynaptic unitary connections when the following criteria were satisfied: (1) all-or-none eIPSCs appearance; (2) absence of increase in eIPSC amplitude when minimal stimulation amplitude was increased by 0.05 mA; (3) disappearance of eIPSCs when stimulation polarity was inverted; and (4) constant latency of the eIPSCs.

Three different interstimulus intervals of stimulation were realized: 20, 50, and 100 ms and were repeated every 3 s. Paired-pulse ratio was determined as the amplitude ratio of the second to the first IPSC evoked in the postsynaptic neuron.

The article "Modulation of GABAergic Synaptic Transmission by NMDA Receptors in the Dorsal Horn of the Spinal Cord" was published in 2022. Journal: Front Mol Neurosci.

### Pharmacological Substances

Different drugs were used in order to study NMDA effects on inhibitory synaptic transmission. We recorded spontaneous IPSCs in the presence of antagonist of AMPA and Kainate receptors, 6-cyano-7-nitroquinoxaline-2,3-dione (CNQX, 10 μM, Tocris). To isolate GABAergic or glycinergic currents, we used strychnine (1 μM, Sigma) or bicuculline methiodine (10 μM, Sigma), respectively. Miniature IPSCs were recorded in the presence of tetrodotoxin (TTX; 0.5 μM, Latoxan) to block voltage gated sodium channels.

To assess the role of NMDAr, we used the specific agonist N-Methyl-D-aspartic acid (NMDA, 100 μM, Tocris). The specific antagonist of NMDAr, D-2-amino-5-phosphonovalerate (APV 50 μM; Abcam), was used to block all NMDAr. Two specific antagonists of NMDAr containing GluN2C/D subunits were used, (2R,3S)-1-[(phenanthren-3-yl)carbonyl]piperazine-2,3-dicarboxylic acid) (UBP141 10 μM and 25 μM) and (4-((1H-Indol-7yl)carbamoyl)phenyl diethylcarbamate) NAB14 (10 μM, from Abcam and Aobious respectively). Ifenprodil (10 μM, Sigma) was used to block NMDAr containing GluN2B subunits. Zinc (100 nM, Sigma) was used to inhibit NMDAr containing GluN2A subunits. Finally, we also used a channel blocker of NMDAr, dizocilpine (MK-801; 2 mM in the intracellular solution, Tocris). Drugs were prepared as 1,000× or 10,000× concentrated stock solutions in dimethylsulphoxide (DMSO), water or ethanol in accordance with indications from the manufacturer. The stocks were stored at −20°C. All substances were diluted to their final concentration in ACSF at the beginning of each experiment and applied by general bath perfusion (flow rate: 1.0 ml/min; total chamber volume: 2 ml).

### Data Analysis

Synaptic events were detected using WinEDR with an amplitude threshold detection algorithm and visually inspected for validity. The analysis of frequency has been performed as described in a previous study of our lab (Petitjean et al., 2012). For each neuron analyzed, the cumulative number, N, of synaptic events was plotted as a function of time. A two-linear-segment curve was fitted by non-linear regression (KyPlot 2.15; KyensLab, Tokyo, Japan) using the following equation:


N=fo×t×a

for t < tc and


N=fc×t+(fo−fc)×tc+a

for t > tc

Where the slope “fo” represents an estimation of the average frequency under control conditions and “fc” provides an estimation of the mean frequency following the application of the drug. “tc” is the time at which the change in frequency occurs. Drugs were considered to have an effect when “tc” occurred around 100 s following the beginning of the application of the substance and when the change in frequency exceeded 20% of the recorded basal frequency.

The article "Modulation of GABAergic Synaptic Transmission by NMDA Receptors in the Dorsal Horn of the Spinal Cord" was published in 2022. Journal: Front Mol Neurosci.

The percentage of increase in frequency was calculated as follows:


$$Change\inf requency\left(\%\right)=\left(\frac{fc-fo}{fo}\right)\times 100$$

Peak amplitude was determined by using WinWCP (waveform measurements) to determine the exact value of the peak. Tau rise and Tau decay were determined by fitting the trace with an exponential decay (EPC endplate current-fitting function of WinWCP) using the following equation:


$$\text{y (t)}=0.5*\text{A}*(1\;+\text{ erf }(\text{x }-\text{ τrise}))*\exp\left(\frac{-\text{x}}{\text{τdecay}}\right)$$

Where A is the amplitude (in pA), τrise is the rise time (in ms) and τdecay is the decay time (in ms). Following these analyses, each neuron was classified either as displaying a change in EPSCs or IPSCs frequency, amplitude or kinetics in response to the application of the substance or as being non-responsive to this substance.

### Statistics

Data are represented as mean ± Standard Error to the Mean (SEM). Statistical analyses were performed with GraphPad Prism (GraphPad Software 6.07, La Jolla, CA, USA). To compare proportions of neurons, Fisher’s exact test was used. For the effect of drug application, we used the paired t-Test or the Wilcoxon test, and the unpaired t-Test or the Mann-Whitney test were used for unpaired comparisons, depending on the data distribution previously tested with the D’Agostino and Pearson normality test.

## Results

### NMDA Receptor Activation Leads to an Increase in Spontaneous GABAergic Synaptic Transmission

Bath application of NMDA (100 μM, 60 s) caused a significant increase in the frequency of spontaneous inhibitory postsynaptic currents (sIPSCs) in 75% of the recorded neurons (*N* = 18/24). This facilitation was always followed by a full recovery after a washout (Figures 1A,B). In neurons displaying a significant increase in sIPSCs frequency, the increase was of 415% (control: 0.19 ± 0.06 Hz, NMDA: 0.79 ± 0.17 Hz; *N* = 18; *t* = 4.147, *p* = 0.0007, paired t-test). In these neurons, increase in sIPSCs frequency occurred without changes in sIPSCs amplitude (control: −32.5 ± 4.0 pA, NMDA: −32.5 ± 4.7 pA; *N* = 18; *t* = 0.003, *p* = 0.9975, paired t-test; Figure 1B).

**Figure 1:** NMDA increases GABA sIPSC frequency in lamina II neurons. **(A)** Representative traces of total sIPSCs recorded from lamina II neuron in spinal cord slice from C57Bl6 mouse before (Control) and during NMDA application (NMDA; 100 s after the beginning of application) and after a washout (wash; 360 s after the beginning of NMDA washout). **(B)** Bar graph showing total sIPSC frequency and peak amplitude before (Control) and during NMDA application (NMDA) and after a washout (wash; *N* = 18). NMDA application resulted in a reversible increase in sIPSC frequency without change in sIPSC amplitude. **(C,D)** Frequency and peak amplitude of GABAergic sIPSCs **(C)** and glycinergic sIPSCs **(D)** isolated pharmacologically. NMDA application enhances GABAergic sIPSC (recorded in presence of strychnine) frequency (*N* = 67) but did not affect glycinergic sIPSCs, recorded in presence of bicuculline **(D)** (*N* = 9). ***p < 0.001. Paired t-test was used. Error bars indicate SEM.

The article "Modulation of GABAergic Synaptic Transmission by NMDA Receptors in the Dorsal Horn of the Spinal Cord" was published in 2022. Journal: Front Mol Neurosci.

Fast synaptic inhibition in the dorsal horn of the spinal cord is mediated by GABA and glycine. Effects of NMDA on GABAergic sIPSCs were examined in presence of 1 μM strychnine, a glycine receptor antagonist and effects of NMDA on Glycinergic sIPSCs were examined in presence of 10 μM bicuculline, a GABA_A_ receptor antagonist. NMDA application induced a reversible increase of GABAergic sIPSCs in 80.7% of the recorded neurons (*N* = 67/83). In neurons displaying a significant effect, NMDA increased GABAergic sIPSCs frequency by 736% (control: 0.11 ± 0.01 Hz, NMDA: 0.81 ± 0.08 Hz; *N* = 67; *t* = 4.147, *p* = 0.0007, paired t-test) without changing sIPCSs amplitude (control: −24.2 ± 1.6 pA, during NMDA: −23.5 ± 1.2 pA; *N* = 67; *t* = 0.9188, paired t-test; Figure 1C). NMDA application neither changed glycinergic sIPSCs frequency nor amplitude (*N* = 9) indicating that NMDA modulates specifically GABAergic synaptic transmission (Figure 1D).

These results indicate that activation of NMDAr increases the frequency of GABAergic and not glycinergic spontaneous IPSCs.

In neurons in which NMDA facilitated GABAergic sIPSCs, a second application of NMDA yielded a similar effect (relative increase in frequency: NMDA = 0.93 ± 0.29, *N* = 6; Figure 2A). Taking advantage of the reproductibility of NMDA effect, we examined the effect of NMDAr antagonists in NMDA-responsive neurons. To this end, a second application of NMDA was performed in presence of NMDAr antagonists or modulators, and effects of both applications were compared.

**Figure 2:** Activation of GluN 2C/D containing NMDA receptors induces increase of spontaneous GABAergic transmission. **(A,B)** Example of the effect of two successive NMDA applications on the number of GABAergic sIPCSs (50 s bin). NMDA effect is reproducible **(A)** and completely blocked in presence of APV (50 μM) **(B)**. **(C)** Effect of a second application of NMDA in presence of different NMDAr selective antagonists. Histogram showing the effect of a second NMDA application normalized to a first application performed in absence of antagonists. NMDA-induced increase in GABA sIPSC frequency was inhibited in presence of APV (50 μM, *N* = 8) and UBP 141 (10 μM, *N* = 4; 25 μM, *N* = 9). Presence of Zinc (100 nM, *N* = 4) or Ifenprodil (10 μM, *N* = 8) did not affect NMDA effect. *p < 0.05 and **p < 0.01. Mann-Whitney test was used. Error bars indicate SEM.

The article "Modulation of GABAergic Synaptic Transmission by NMDA Receptors in the Dorsal Horn of the Spinal Cord" was published in 2022. Journal: Front Mol Neurosci.

In the presence of 50 μM APV, a selective NMDAr antagonist, NMDA-induced increase in GABAergic sIPSCs frequency was reduced by 72% (relative increase in frequency: NMDA = 0.93 ± 0.29, NMDA+APV = 0.28 ± 0.07, *N* = 8, *p* = 0.02, Mann-Whitney test; Figure 2B).

NMDAr is a tetrameric ionotropic glutamate receptor with a most frequent configuration consisting of two mandatory GluN1 and two GluN2 subunits (GluN2 A-D). To assess the composition of NMDAr contributing to the increase in GABAergic sIPSCs frequency, we tested the effect of NMDAr subunit-selective antagonists.

Zinc (100 nM), which blocks specifically NMDAr containing GluN2A subunit, had no effect on NMDA-induced effect (relative increase in frequency: Zinc = 1.40 ± 0.30, *N* = 4), neither did ifenprodil (10 μM), a selective antagonist of GluN2B-containing NMDAr (relative increase in frequency: ifenprodil = 0.94 ± 0.25, *N* = 8). However, NMDA-induced increase in GABAergic sIPSCs frequency was reduced by 79% in presence of UBP 141 (UBP 10 μM: relative increase in frequency = 0.21 ± 0.08, *N* = 4, *p* = 0.019, Mann-Whitney test; UBP 25 μM: relative increase in frequency = 0.20 ± 0.04, *N* = 9, *p* = 0.0048, Mann-Whitney test) a specific antagonist of GluN2C/D-containing NMDAr (Figure 2C), indicating the involvement of NMDAr containing these subunits in the effects of NMDA on GABAergic transmission.

### NMDA Receptor Activation Selectively Increases GABA Release

We next examined whether NMDA-induced facilitation of spontaneous GABAergic transmission involved a direct effect on presynaptic GABAergic terminals or whether it required action potential firing and propagation in presynaptic interneurons. To this end, we recorded miniature IPSCs (mIPSCs) in the presence of 0.5 μM TTX. In 58% of recorded-neurons (*N* = 14/24), application of NMDA induced a significant increase in mIPSCs frequency (control: 0.04 ± 0.01 Hz, NMDA: 0.21 ± 0.05 Hz; *N* = 14; *t* = 3.664, *p* = 0.0029, paired t-test), without change in mIPSCs amplitude. We next recorded pharmacologically isolated GABAergic mIPSCs in the presence of the channel blocker TTX and the glycine receptor antagonist Strychnine (STR). In 54% of recorded neurons (*N* = 35/65), NMDA induced a significant increase in GABAergic mIPSCs frequency (control: 0.07 ± 0.01 Hz, NMDA: 0.26 ± 0.04 Hz; *N* = 36; *t* = 5.364, *p* < 0.0001, paired t-test) without changes in GABAergic mIPSCs amplitude (Figures 3A,B). Moreover, NMDA never induced significant changes neither in amplitude, nor in mIPSCs activation or deactivation kinetics, suggesting that NMDA increased GABA release probability *via* a presynaptic action.

The article "Modulation of GABAergic Synaptic Transmission by NMDA Receptors in the Dorsal Horn of the Spinal Cord" was published in 2022. Journal: Front Mol Neurosci.

**Figure 3:** Activation of GluN2C/D containing NMDA receptor increase miniature GABAergic IPSCs. **(A)** Representative traces of mIPSCs recorded from a lamina II neuron in spinal cord slice from C57Bl6 mouse before (Control) during NMDA application (NMDA; 100 s after the beginning of application) and after a washout (wash; 400 s after the beginning of NMDA washout). **(B)** Bar graph showing total mIPSC (*N* = 14) and GABA mIPSC (*N* = 36) frequency and peak amplitude before (Control) and during NMDA application (NMDA). **(C)** Effect of APV (50 μM, *N* = 6) and NAB 14 (10 μM, *N* = 5) on NMDA-induced increase in GABA mIPSC frequency. Both antagonists blocked effect of NMDA application. **(D)** NMDA-induced increase in GABA mIPSC frequency in presence (2 mM Mg^2+^, *N* = 36) or in absence of external Mg^2+^ (0 mM Mg^2+^, *N* = 5) is comparable. *p < 0.05, **p < 0.01, ***p < 0.001. Paired t-test **(A)**, Mann-Whitney test **(B)**, and Wilcoxon test **(C)** were used. Error bars indicate SEM.

To examine the specificity of the NMDA effect on GABAergic synapses, we examined the effect of NMDA application on mEPSCs or glycinergic mIPSCs. NMDA applications neither changed mEPSCs (recorded without CNQX and in presence of bicuculline and strychnine), nor glycinergic mIPSCs (recorded in absence of Strychnine and in presence of CNQX and bicuculline; data not shown).

As previously performed for spontaneous GABAergic transmission, we observed the effects of NMDAr antagonists on the NMDA-induced increase in mIPSCs frequency.

APV (50 μM) reduced by 72% the NMDA-induced increase in GABAergic mIPSCs frequency (relative response to the first application: NMDA = 0.59 ± 0.11, APV = 0.17 ± 0.04, *N* = 6, *p* = 0.0087, Mann-Whitney test; Figure 2B). These results confirm that NMDA acted on NMDAr to increase the frequency of GABAergic mIPSCs.

NMDA-induced increase in GABAergic mIPSCs frequency was reduced by 77% in presence of NAB14 (10 μM) a highly selective antagonist of GluN2C/D-containing NMDAr (relative response: NAB14 = 0.23 ± 0.05, *N* = 5, *p* = 0.0173, Mann-Whitney test) confirming the involvement of GluN2C/D-containing NMDAr in NMDA-induced facilitation of GABAergic synaptic transmission (Figure 3C).

The voltage-dependent block of NMDAr by Mg^2+^ is stronger for NMDAr containing GluN2A or GluN2B subunits than for those containing GluN2C/D subunit (Paoletti et al., 2013). The experiments described so far were performed in the presence of 2 mM Mg^2+^. To assess whether the contribution of GluN2A- or GluN2B-containing NMDAr was masked by a Mg^2+^-dependent block, we assessed the effect of NMDA on GABAergic mIPSCs recorded in absence of extracellular Mg^2+^. These recordings were performed in presence of MK801 (2 mM) in the recording pipette in order to prevent activation of NMDAr present on the recorded neuron. The stimulatory effect of NMDA on GABAergic mIPSCs was unchanged under these conditions. In 50% of the recorded cells (*N* = 5/10) NMDA application induced an increase in frequency of GABAergic mIPSCs (control: 0.10 ± 0.07 Hz, during NMDA: 0.34 ± 0.08 Hz; *N* = 5; *p* = 0.0625, Wilcoxon test) without any change in mIPSCs amplitude (data not shown; Figure 3D).

The article "Modulation of GABAergic Synaptic Transmission by NMDA Receptors in the Dorsal Horn of the Spinal Cord" was published in 2022. Journal: Front Mol Neurosci.

### NMDAr-Dependent Modulation of GABAergic Transmission Depends on the Neurochemical Identity of the Postsynaptic Neuron

The NMDA-induced increase in GABAergic IPSCs frequency was only observed in 80.7% (spontaneous IPSC) and 54.0% (miniature IPSC) of recorded neurons. We therefore wondered whether NMDA-induced facilitation of GABAergic transmission would depend on the excitatory or inhibitory phenotype of the postsynaptic neurons (from which we recorded). To this end, we perfrormed recordings using slices prepared from GAD65-eGFP mice.

NMDA increased the frequency of spontaneous GABAergic IPSCs recorded both in eGFP+ and eGFP-, in similar proportions (eGFP+: 100%, *N* = 10/10; eGFP-: 85% *N* = 6/7). These results were similar to those obtained from C57Bl6 mice (Figure 4A).

**Figure 4:** NMDA enhancement of mIPSC frequency target specifically GABAergic interneurons. **(A)** Proportion of recorded neurons showing an increase of GABA sIPCS frequency by NMDA application, in unidentified neurons from C57bl6 mice and GAD positive (GAD+) or GAD negative (GAD-) neurons from GAD65-eGFP mice. **(B)** Proportion of recorded neurons recorded showing an increase of GABA mIPCS frequency by NMDA application is significantly higher in GAD positive (GAD+) neurons than for GAD negative (GAD-). **(C,D)** Frequency **(C)** and peak amplitude **(D)** of GABAergic mIPSCs recorded in GAD+ and GAD- neurons from GAD65-eGFP mice. Effect of NMDA on mIPSC frequency is independent of the neuron type. ***p < 0.001. Fischer’s exact test **(B)** and Paired t-test **(C)** were used. Error bars indicate SEM.

A large majority of eGFP+ neurons displayed a facilitatory effect of NMDA on GABAergic mIPSCs (91%, *N* = 20/22). However, a significantly lower proportion of eGFP- neurons (22%, *N* = 2/9, *p* = 0.00042, Fischer’s exact test) showed an effect of NMDA on GABAergic mIPSCs (Figure 4B). As previously observed in “unidentified” neurons, NMDA application increased GABAergic mIPSCs frequency (control: 0.07 ± 0.02 Hz, during NMDA: 0.25 ± 0.05 Hz; *N* = 20; *t* = 4.880, *p* = 0.0001, paired t-test) but neither change in mIPSC amplitude (control: −17.5 ± 1.3 pA, during NMDA: −16.8 ± 1.4 pA; *N* = 20; *t* = 0.5017, paired t-test) nor kinetics (data not shown; Figures 4C,D). In eGFP- neurons displaying an effect, NMDA application also increased GABAergic mIPSCs frequency (control: 0.10 ± 0.04 Hz, during NMDA: 0.21 ± 0.07 Hz; *N* = 2; Figure 4C). These results indicate that the facilitation of GABAergic synaptic transmission by presynaptic NMDAr depends on the postsynaptic target: it preferentially occurs in GABAergic connections onto eGFP+ neurons.

The article "Modulation of GABAergic Synaptic Transmission by NMDA Receptors in the Dorsal Horn of the Spinal Cord" was published in 2022. Journal: Front Mol Neurosci.

### NMDA Changes the Paired-Pulse Ratio and Inhibits Evoked GABAergic IPSCs

An increase in mIPSCs frequency with no change in amplitude suggested a presynaptic mechanism of action of NMDA. We further tested this possibility by determining the effect of NMDA on the paired-pulse ratio (PPR) of electrically-evoked IPSCs (eIPSCs) in eGFP+ neurons (Figure 5A). The relative change in absolute PPR was consistently different from 0 at all interpusle interval tested: 20 ms interpulse (ΔPPR = 0.19 ± 0.07, *N* = 8, *t* = 2.751, *p* = 0.0285, one sample t-test), 50 ms interpulse (ΔPPR = 0.19 ± 0.06, *N* = 9, *t* = 3, *p* = 0.0112, one sample t-test) or 100 ms interpulse (ΔPPR = 0.19 ± 0.07, *N* = 9, *t* = 0.1944, *p* = 0.0205, one sample t-test; Figure 5B).

**Figure 5:** NMDA inhibits evoked IPSCs in GAD-eGFP positive neurons. **(A)** Average of 10 traces representing the response to two successive stimulations separated by 50 ms before (black, control) and during NMDA application (orange, NMDA) and after a washout (gray, wash). **(B)** Histograms showing the relative change in PPR measured in GAD positive cells, for three different paired stimulation interval: 20 ms (*N* = 8), 50 ms (*N* = 9), and 100 ms (*N* = 9). **(C)** Time course of normalized GABAergic eIPSC amplitude before and after NMDA application (*N* = 17). **(D)** Histogram showing average eIPSC amplitude before (control) NMDA application, after NMDA application (NMDA) and after a washout (wash; *N* = 17). *p < 0.05 and ***p < 0.001. One sample t-test **(B)** and paired t-test **(D)** were used. Error bars indicate SEM.

In these neurons, NMDA reduced the mean amplitude of eIPSCs (control: −37.5 ± 3.9 pA, during NMDA: −24.7 ± 2.6 pA; *N* = 17; *t* = 6.029, *p* < 0.0001, paired t-test). This inhibition remains significant at least during 5 min following NMDA washout (Wash −24.4 ± 2.6 pA, *N* = 17, compared to control *t* = 2.440, *p* = 0.0267, paired t-test; Figures 5C,D). These results are consistent with a NMDAr-mediated shunt of action potential dependent release of GABA and confirm that NMDAr modulate GABAergic transmission by a presynaptic mechanism of action.

The article "Modulation of GABAergic Synaptic Transmission by NMDA Receptors in the Dorsal Horn of the Spinal Cord" was published in 2022. Journal: Front Mol Neurosci.

## Discussion

Our results show that activation of NMDAr containing GluN2C/D subunits increased the frequency of GABAergic spontaneous and miniature IPSCs in lamina II neurons. Furthermore, this facilitation of spontaneous and miniature GABAergic IPSCs by NMDAr was preferentially observed for GABAergic connections onto eGFP+ neurons. Interestingly, NMDAr activation reduced the amplitude of electrically-evoked IPSCs recorded.

### NMDAr Subunit Composition and Mg^2+^ Sensitivity

NMDAr are abundant in the dorsal horn with GluN1 and GluN2A/B receptors subunits expressed virtually in all lamina I and II neurons (Nagy et al., 2004). Concerning GluN2C/D subunits, their level of expression is lower in the dorsal horn compared to other GluN2 subunits. But it has been shown that GABAergic interneurons also express NMDAr containing GluN2C/D subunits. These receptors may play a role in modulating the activity of inhibitory interneurons in the dorsal horn of the spinal cord (Shiokawa et al., 2010). Recently, a sex-specific expression pattern of GluN2D subunit has been reported in young rats (P21), with a larger expression of this subunit in male compared to female in superficial regions of the dorsal horn (Temi et al., 2021). We used only male mice in our study; therefore, the modulation of the GABAergic synaptic transmission by NMDAr activation could be different in female mice and would require further investigation.

Using a pharmacological approach, we identify GluN2C/D containing NMDAr as responsible for the NMDA-induced increase of spontaneous GABA release. The increase in mIPSC frequency was comparable in the presence of 2 mM Mg^2+^ or in the absence of Mg2+ indicating low sensitivity to Mg^2+^ block of the NMDAr. This is in agreement with the fact that the presence of GluN2C/D subunits reduces the voltage-sensitive Mg^2+^ block of NMDAr and therefore allows an activation by endogenous glutamate even without depolarization to relieve the Mg^2+^ block (Paoletti, 2011). These properties of NMDAr are well suited for a presynaptic NMDAr function because it may allow receptors to sense level of ambient glutamate and to be activated in the absence of depolarization, and thus under resting conditions. Inhibition may be thus finely regulated according to the overall level of glutamate and to the excitatory activity in the network (Bouvier et al., 2015).

### NMDA Receptor Localization

In the superficial laminae of the dorsal horn, NMDAr are present in virtually every excitatory synapse and therefore in every interneuron (Nagy et al., 2004). NMDA receptors have also been immunocytochemically detected on presynaptic terminals of primary afferents (Liu et al., 1994; Lu et al., 2003) where they regulate neurotransmitter release from the terminals of primary afferent neurons (Bardoni, 2013). Presynaptic localization of NMDAr on GABAergic terminals is less documented. Only one immunohistochemical study has reported that, NMDArs are present on a subset of GABAergic terminals (37%) in rat superficial dorsal horn (Lu et al., 2005); however, the role of these receptors has not been investigated so far.

The article "Modulation of GABAergic Synaptic Transmission by NMDA Receptors in the Dorsal Horn of the Spinal Cord" was published in 2022. Journal: Front Mol Neurosci.

In other regions of the CNS, such as cerebellum, neocortex, prefrontal cortex, and visual cortex, immunocytochemical and functional studies have documented the presence of presynaptic NMDAr involved in modulation of GABA release (Glitsch and Marty, 1999; Mathew and Hablitz, 2011; Abrahamsson et al., 2017; Pafundo et al., 2018). Some of these studies reported a differential regulation of evoked and spontaneous release by presynaptic NMDAr (Glitsch and Marty, 1999; Abrahamsson et al., 2017) comparable with our results. Indeed, we showed that NMDA increased the frequency of GABAergic mIPSCs but depressed evoked GABAergic IPSCs recorded in lamina II neurons. Considering a presynaptic localization, NMDAr activation could induce a calcium influx through the NMDAr channel, and thereby facilitate synaptic vesicle exocytosis and spontaneous GABA release. The same presynaptic NMDAr could depress evoked GABA release by decreasing the input resistance, thereby shunting the propagation of incoming action potentials. Presynaptic NMDAr could also depolarize synaptic boutons, inactivate voltage gated Na^+^ channels and elevate the threshold for action potential generation. Both mechanisms would result in an increase in transmission failure and a reduction of the probability of evoked GABA release. Finally, presynaptic NMDAr could act *via* distinct and independent pathways to control evoked and spontaneous release separately as recently shown in the visual cortex (Abrahamsson et al., 2017).

However, our results provide indirect evidence for a presynaptic localization of NMDAr with important limitations. We cannot exclude that NMDAr are expressed near the GABAergic synapse and that NMDA might act by an indirect effect implicating a second messenger. Indeed, postsynaptic NMDAr activation could be the source of calcium needed to trigger and/or release a retrograde messenger such as NO. For example, NO could act retrogradely on the presynaptic terminal and facilitate GABA release. Such a mechanism has been reported in the dorsal horn were NO release was triggered by metabotropic glutamate receptor (mGluR1) activation and induced a heterosynaptic LTP of GABAeric synapses (Fenselau et al., 2011). Interestingly, in the dorsal horn, NO synthase is expressed in 17% of GABAergic interneurons (Boyle et al., 2017) and we found that NMDAr-dependent modulation of GABAergic transmission targeted preferentially inputs to GABAergic neurons. However, this mechanism could only explain the facilitatory effect observed on spontaneous transmission but not the depression of evoked IPSCs.

The article "Modulation of GABAergic Synaptic Transmission by NMDA Receptors in the Dorsal Horn of the Spinal Cord" was published in 2022. Journal: Front Mol Neurosci.

Finally, recent investigations have shown that functional NMDAr were present on astrocytes (Ziak et al., 1998; Lalo et al., 2006; Palygin et al., 2011), and activation of these astroglial NMDAr is involved in neuron-to-glia communication, and in the modulation of inhibitory synaptic transmission (Lalo et al., 2006, 2014). Such astroglial receptors could be involved in our results but once again could not completely explain the differential modulation of spontaneous and evoked GABA release.

However implication of different NMDAr with different localizations can drive bidirectional plasticities at GABAergic synapses (Mapelli et al., 2016) and thus could explain the differential regulation of GABAergic transmission that we observed.

In our experiments, the frequency of glycinergic mIPSCs was unaffected, indicating that presynaptic modulation of inhibitory synaptic transmission by NMDAr activation was exclusively observed at GABAergic nerve terminals and selectively controlled spontaneous GABAergic synaptic transmission. These results are in accordance with a recent study by Kloc and collaborators who showed that NMDAr activation induced LTP at glycinergic synapses that depended upon an increase in the number and/or the properties of Glycinergic receptors but was independent of glycine release (Kloc et al., 2019). In the DH, most dorsal horn neurons receive both GABAergic and glycinergic inputs, but these inputs may arise from neurons having their cell body localized in distinct laminae. Inhibitory interneurons in lamina II are virtually only GABAergic since glycinergic cell bodies were almost absent in this lamina (Zeilhofer et al., 2005; Punnakkal et al., 2014). A selective modulation of GABAergic transmission by NMDAr might therefore correspond to a restricted modulation of inhibition within lamina II processing nociceptive information.

Physiologically, glutamate required to activate NMDAr responsible for GABAergic synapse modulation may originate from neighboring excitatory synapses. In this case, NMDAr activation would depend on glutamate diffusion from neighboring synapses as previously described in the cerebellum (Huang and Bordey, 2004; Duguid and Smart, 2009). In the dorsal neuronal horn network ambient levels of glutamate are tightly regulated by glutamate transporters. These transporters (mainly expressed by glial cells) have a crucial role in limiting glutamate diffusion and crosstalk between neighboring synapses. Interestingly, in pathological states such as during neuropathic pain induced by a nerve injury, disruption of glutamate homeostasis in the DH led to an increase in extracellular levels of glutamate and subsequent spillover (Inquimbert et al., 2012). Therefore the modulation of GABAergic synaptic transmission by NMDA receptors we described in this study could be a new spinal mechanism involved in the development of neuropathic pain. Moreover, subunit composition and properties of NMDAr are altered by inflammation and peripheral nerve injury (Guo and Huang, 2001; Iwata et al., 2007) and consequently the modulation of GABAergic transmission by NMDAr activation could be modified.

The article "Modulation of GABAergic Synaptic Transmission by NMDA Receptors in the Dorsal Horn of the Spinal Cord" was published in 2022. Journal: Front Mol Neurosci.

Altogether our results strongly suggest that glutamate can directly activate GluN2C/D containing NMDAr which differentially regulate GABA release. This crosstalk between excitation and inhibition could control the excitation/inhibition balance in the spinal neuronal network. It will be critical in future work to clarify the localization of NMDAr involved in the regulation of GABAergic transmission targeting GABAergic neurons and to define their role in the processing of nociceptive information in spinal neuronal network in physiological, inflammatory and neuropathic pain conditions.

## Data Availability Statement

The original contributions presented in the study are included in the article, further inquiries can be directed to the corresponding author.

## Ethics Statement

The animal study was reviewed and approved by Regional ethics committee and the French Ministry of Agriculture.

## Author Contributions

BL, LC, and LV-M performed acquisition and analysis of data. This study was designed by PI, SH, and RS. The manuscript was written by PI, SH, RS, and BL. All authors contributed to the article and approved the submitted version.

## Conflict of Interest

The authors declare that the research was conducted in the absence of any commercial or financial relationships that could be construed as a potential conflict of interest.

## Publisher’s Note

All claims expressed in this article are solely those of the authors and do not necessarily represent those of their affiliated organizations, or those of the publisher, the editors and the reviewers. Any product that may be evaluated in this article, or claim that may be made by its manufacturer, is not guaranteed or endorsed by the publisher.
